# Neoadjuvant Chemotherapy plus Bevacizumab Combined with Total Mesorectal Excision in Treating Locally Advanced Rectal Cancer Patients with BRAF Mutation: Clinical Benefit and Safety

**DOI:** 10.1155/2021/4227650

**Published:** 2021-12-09

**Authors:** Jintian Song, Yi Wang, Hui Yu, Liang Zheng, Xiongchao Cai, Yigui Chen

**Affiliations:** ^1^Department of Abdominal Oncology, Fujian Medical University Cancer Hospital, Fujian Cancer Hospital, Fuzhou City, Fujian Province 350014, China; ^2^Department of Abdominal Tumor Surgery, Fujian Medical University Cancer Hospital, Fujian Cancer Hospital, Fuzhou City, Fujian Province 350014, China; ^3^Department of Pharmacy, Fujian Medical University Cancer Hospital, Fujian Cancer Hospital, Fuzhou City, Fujian Province 350014, China

## Abstract

**Objective:**

To investigate clinical benefit and safety of neoadjuvant chemotherapy (NAC) plus bevacizumab combined with total mesorectal excision (TME) in treating patients with BRAF-mutated locally advanced rectal cancer (LARC).

**Methods:**

This study included LARC patients with BRAF mutation admitted to the Oncology Department of Fujian Medical University Cancer Hospital, Fujian Cancer Hospital, between June 2013 and December 2018. Patients in the control group received a standard treatment regimen of TME combined with NAC (*n* = 45), and patients in the observation group received NAC plus bevacizumab combined with TME (*n* = 55). The short-term clinical efficacy of the two groups after NAC treatment was observed and compared, including differences in the pathological downstaging rate. The incidence of perioperative complications and adverse reactions during neoadjuvant therapy was compared to evaluate the safety of the treatment. Besides, the relapse-free survival (RFS) and overall survival (OS) of patients were analyzed to evaluate the long-term clinical benefit of the treatment.

**Results:**

Compared with the control group, the ypT staging rate (*p* = 0.014) in the observation group was markedly lower. In addition, patients in the observation group had a prominently lower overall incidence of complications (*p* < 0.001) during the perioperative period and a remarkably lower incidence of leukopenia (*p* = 0.037) during neoadjuvant therapy. In terms of long-term clinical benefit, the RFS of patients in the observation group was evidently longer (*p* = 0.037) than that in the control group.

**Conclusion:**

Compared with TME plus NAC treatment, the short-term and long-term clinical benefits are higher and safety is more favorable of NAC plus bevacizumab combined with TME in treating LARC patients.

## 1. Introduction

The clinical diagnosis and treatment of rectal cancer have always been challenging medical problems due to high difficulty in operation and high local relapse rate. Neoadjuvant chemoradiotherapy (NCRT) combined with total mesorectal excision (TME) is a standard clinical treatment for locally advanced rectal cancer (LARC) [1]. Clinical studies indicated that no tumor cells were detected in postoperative pathological tissue in about 20% of LARC patients who received TME after NCRT, suggesting a pathological complete response (pCR) [2]. However, many clinical studies reported that this standard treatment method deficits in two main aspects. Although it can reduce the local relapse rate of patients, evident survival benefits were not achieved in terms of long-term efficacy [3, 4]. In addition, due to the high damage of radiotherapy to LARC patients, anal function, urination function, and sexual function worsen with time, which dramatically reduces the patient's life quality and increases the risk for secondary tumors such as bladder cancer [5–7]. With the continuous development of TME-related techniques in clinical practice, both the R0 resection rate and anus preservation rate are becoming more and more ideal. At present, the most vital risk factor for LARC mortality is distant metastasis. It is also becoming increasingly crucial to treat patients with systemic chemoradiotherapy. However, radiotherapy will lead to decreased compliance of LARC patients with postoperative adjuvant chemotherapy after TME, which may be the cause of poor prognosis in some patients [8–10]. Hence, neoadjuvant chemotherapy (NAC) has become another popular choice for LARC treatment in recent years. All LARC patients included in this study did not receive preoperative radiotherapy, and NAC was utilized as the primary treatment strategy before TME.

In recent years, studies have shown that gene mutations in cancer patients are prominently related to their prognosis. For example, BRAF mutation has been proven to be a vital factor affecting chemotherapeutic resistance and survival rate of colorectal cancer and non-small-cell lung cancer [11, 12]. The treatment of BRAF-mutated LARC has always been a hot and difficult topic. With the continuous development of clinical drug and the enrichment of clinical data, some scholars proposed that in patients who harbor BRAF-mutated tumors, the antiangiogenic therapy of bevacizumab combined with chemotherapy is effective and the clinical value of bevacizumab is much higher than that of cetuximab [13]. However, at present, there are few clinical studies on the use of NAC plus bevacizumab in LARC patients with BRAF mutation.

Bevacizumab is a type of drug that targets the vascular endothelial growth factor receptor and has been proven to show clinical therapeutic effect in multiple tumors [14]. In the clinical treatment for rectal cancer, this drug can be employed in combination with chemotherapeutic drugs to facilitate the sensitivity of patients, which is conductive to improving the efficacy of chemotherapy and thereby improving the overall survival rate of patients [15, 16]. Schrag et al. [17] conducted a prospective study on 32 LARC patients and added bevacizumab to NAC to explore the R0 resection rate of TME and the pCR rate of patients. Finally, it was confirmed that the neoadjuvant treatment of NAC plus bevacizumab has good safety and the patient's survival conditions are also ideal. Another meta-analysis also reached a similar conclusion, supporting that the addition of bevacizumab in NAC has ideal safety while improving the efficacy [18]. In summary, adding bevacizumab to NAC may be a safe and feasible preoperative option for neoadjuvant therapy in LARC. As a result, in this retrospective study, we chose to explore the clinical efficacy and safety of bevacizumab in combination with NAC.

Taken together, we speculated that NAC plus bevacizumab treatment combined with TME for LARC patients with BRAF mutation may achieve better clinical efficacy, and we explored it in this study. By collecting BRAF-mutated LARC patients who received NAC with or without bevacizumab combined with TME treatment, we evaluated the short-term and long-term clinical benefits of patients after receiving treatment.

## 2. Methods

### 2.1. Sample Collection and Grouping

The subjects of this study were LARC patients, and the diagnostic criteria were as follow: the primary tumor found by imaging or pathological examination invades the muscular layer of the intestinal wall to the surrounding structures (c/pT3-4) or develops lymph node metastasis (c/pN1-2) without distant metastasis (M0) in the mesangium and true pelvis within 12 cm from the anus. The aforementioned LARC patients were admitted to the oncology department of our hospital from June 2013 to December 2018. The BRAF mutation of the patients was detected to confirm that the LARC patients had BRAF mutation. Patients were then divided into the observation group and control group according to the treatment regimen. LARC patients in the observation group received NAC plus bevacizumab followed by TME (*n* = 55), and the control group was LARC patients receiving NAC followed by TME (*n* = 45). The baseline data of the patients at the time of admission are shown in Table 1. The tumor status was evaluated by the TNM staging system of the eighth edition of the American Joint Committee on Cancer (AJCC) [19]. There was no evident difference in the baseline data of LARC patients between the observation group and the control group.

### 2.2. Detailed Treatment Plan

Liver-protective drugs, antiemetic drugs, and dexamethasone for allergy prevention and hydration therapy were routinely utilized in all patients during NAC.

All patients received preoperative NAC. Drugs and dosage regimen used were as follows: oxaliplatin (manufacturer: Jiangsu Hengrui Pharmaceutical Co., Ltd.; approval no.: national medicine permission number H20000337; specifications: 50 mg), 130 mg/m^2^ intravenously administered for 2 h on day 1 of each course, and capecitabine (manufacturer: Jiangsu Hengrui Pharmaceutical Co., Ltd.; approval number: national medicine permission number H20133366; specifications: 0.15 g), 1000 mg/m^2^ oral administration on day 1 to day 14 of each course. Three weeks of NAC were defined as one course of treatment.

Patients in the observation group were given bevacizumab during NAC treatment. The manufacturer of bevacizumab was Roche Diagnostics GmbH, Roche Pharma (Schweiz) Ltd. approval no.: S20170035; specifications: 100 mg (4 mL)/vial. Bevacizumab (5 mg/kg) was given in intravenous infusion for 30 min on day 1 of each course, and every 3 weeks were defined as one course of treatment.

Except for the patients realizing pCR during NAC, the rest received TME at an interval of 5-12 weeks after NAC. All the patients received conventional postoperative adjuvant chemotherapy according to the disease progression.

### 2.3. Observation Indexes of Short-Term Clinical Benefit

The short-term clinical benefit of the two groups of patients after receiving treatment, complications of TME perioperative patients, short-term efficacy of NAC with bevacizumab, and anus preservation rate of TME were recorded and compared.

After TME, the excised pathological tissue was collected and the tumors in the tissue specimens were detected. The TNM staging system of the eighth edition of AJCC was also employed to evaluate the therapy pathological TNM (ypTNM) of patients after the preoperative treatment to analyze downstaging.

The R0 resection rate and perioperative complications of LARC patients were compared between the observation group and the control group, including anastomotic leakage, early postoperative intestinal obstruction, incision infection dehiscence, urinary retention, and anastomotic bleeding.

The incidence of adverse reactions during neoadjuvant therapy of LARC patients between the observation group and the control group was compared, including bone marrow suppression, gastrointestinal reactions, neurotoxic effects, leukopenia, and impaired liver and kidney function.

### 2.4. Observation Indicators of Long-Term Clinical Benefit

The follow-up data of the patients included in this study were collected, and the patients' RFS and OS were utilized as indicators to evaluate long-term clinical benefit. Among them, RFS was the main outcome event of long-term clinical benefit, which was defined as the time from the patient's diagnosis to the patient's tumor relapse or the end of follow-up due to any reason. OS was a secondary outcome event of long-term clinical benefit, which was defined as the time from the diagnosis of the patient to the death by any cause or the end of follow-up due to any cause.

### 2.5. Statistical Analysis

In this study, SPSS 26.0 software was applied for the statistical analysis process. Fisher's exact test or chi-square test was adopted for categorical variables. Continuity variables were tested for normality and homogeneity of variance. Continuous variables conforming to normal distribution were expressed in the form of mean ± standard deviation, and a two-sided *t*-test was utilized to statistically analyze the differences between the data. The continuous variables with skewed distribution were expressed in the form of median (interquartile range), and the Mann-Whitney *U* test was used for testing. The Kaplan-Meier method was applied to analyze the patients' RFS and OS, and the log-rank test was employed to compare the differences between the two groups of data. *p* < 0.05 indicated that the difference was prominent, which was statistically significant.

## 3. Results

### 3.1. Short-Term Efficacy Comparison

Overall, there was no significant difference between total T downstaging (8) and total N downstaging (*p* = 0.813) between the two groups, but difference in ypT staging distribution (*p* = 0.014) between the two groups was statistically significant (Table 2).

### 3.2. Clinical Safety Analysis

In this section, we mainly compared the perioperative complications of BRAF-mutated LARC patients who received TME, the R0 resection rate of TME, and the incidence of adverse reactions during chemotherapy in two groups, so as to explore the effect of adding bevacizumab to NAC on the safety of clinical treatment. In terms of the safety of TME, all patients in this study achieved R0 resection for the first TME, and the complications are shown in Table 3. The incidence of anastomotic leakage (*p* = 0.135), early postoperative intestinal obstruction (*p* = 0.171), incision infection dehiscence (*p* = 0.061), urinary retention (*p* = 0.655), and anastomotic bleeding (*p* = 0.655) in the observation group during the perioperative period was higher than that in the control group, without evident difference. There were marked differences in the overall incidence of complications (*p* < 0.001). Secondly, by comparing the incidence of adverse reactions in the two groups of patients during neoadjuvant therapy, we uncovered that there were differences in the incidence of adverse reactions between the two groups of patients. The incidence of bone marrow suppression (*p* = 0.179), gastrointestinal reactions (*p* = 0.228), neurotoxicity (*p* = 0.090), leukopenia (*p* = 0.037), and liver and kidney damage (*p* = 0.361) in the observation group was lower than that in the control group, and the incidence of leukopenia in the observation group was reduced markedly (Table 4).

### 3.3. Long-Term Efficacy Comparison

In this section, the survival of the two groups of patients was compared, and the long-term clinical benefit in LARC patients with BRAF mutation receiving NAC plus bevacizumab followed by TME was evaluated. After comparing the RFS of the two groups of patients, it was revealed that there were prominent differences in the RFS between the two groups (*p* = 0.037): the median RFS time of LARC patients in the observation group was 27.6 months while in the control group, it was 25.9 months. The RFS in the observation group was markedly longer than that in the control group (Figure 1(a)). By comparing the OS of the two groups of patients, it was uncovered that there was no evident difference (*p* = 0.207) in OS between the two groups. The median OS time of LARC patients in the observation group was 28.9 months, and that of the control group was 27.7 months. There was no prominent difference in OS between the two groups (Figure 1(b)).

## 4. Discussion

NAC refers to the method of systemic chemotherapy on patients before surgery to improve their tumor condition and prepare for later surgery by preoperative chemotherapy. It was proven to be effective in reducing the tumor stage, shrinking the tumor, and improving the surgical success rate in various malignant tumors such as breast cancer and bladder cancer [20, 21]. At present, the clinical benefit of NAC followed by TME in LARC is also a crucial issue of medical attention. In addition, a recent study proved that the addition of bevacizumab to NAC shows good efficacy and safety in the clinical treatment of ovarian cancer, and this method also has a good research prospect in other tumors [22]. BRAF mutation has been proven to predict the efficacy of targeted drugs in the treatment of colorectal cancer and is an independent negative factor affecting the clinical efficacy of bevacizumab added to chemotherapy [23, 24]. Hence, this study included LARC patients with BRAF mutation. By comparing the clinical short-term and long-term effects of bevacizumab on NAC combined with TME treatment, the value of bevacizumab in the clinical treatment of BRAF-mutated LARC patients was explored.

This study showed that LARC patients in the observation group who received NAC plus bevacizumab expressed excellent clinical efficacy in many aspects. In this study, we compared the OS and RFS in the observation group and the control group and confirmed that after adding bevacizumab to NAC, the RFS of LARC patients was prominently prolonged. It was shown that the addition of bevacizumab to NAC greatly improved the long-term clinical benefit. In addition, by comparing the complications of TME and the incidence of adverse reactions during chemotherapy between the two groups of patients, it was revealed that bevacizumab played a positive part in the safety of the treatment and prominently reduced the overall incidence of perioperative complications and the incidence of leukopenia during chemotherapy. The short-term clinical benefit of NAC plus bevacizumab was evaluated by comparing the patient's pathological downstaging after treatment. It was uncovered that compared with the control group, the observation group had a prominently lower T downstaging rate. The above results all indicated that the addition of bevacizumab to NAC was markedly related to better short-term clinical benefit. Similarly, in a clinical study involving 70 patients with colorectal cancer, it was revealed that the addition of bevacizumab to the NAC produced a good objective response rate, clinical benefit rate, R0 resection rate, and acceptable incidence of adverse reactions. It was indicated that NAC plus bevacizumab is a safe and effective treatment strategy that can improve the life quality of patients [25].

Overall, this study confirmed the value of adding bevacizumab to NAC to treat patients with BRAF-mutated LARC. After the addition of bevacizumab, the clinical treatment displayed better short-term and long-term clinical benefits and higher safety. Therefore, bevacizumab can be added to NAC to achieve a more ideal therapeutic effect on BRAF-mutated LARC patients receiving standard treatment.

This study is subject to certain limitations. Due to the small number of patients included in this study, whether this conclusion has the value for large-scale clinical promotion still needs in-depth research. Besides, we did not conduct subgroup survival analysis of the two groups; therefore, we failed to discuss what other clinical factors can affect the prognosis of patients in addition to therapeutic strategies. More clinicopathological data of LARC patients with BRAF mutations and clinical risk factors affecting the patient's prognosis would contribute to the improvement of the LARC patient's prognosis.

## Figures and Tables

**Figure 1:** RFS and OS curves of LARC patients in the observation group and the control group: (a) RFS survival curve of the two groups of patients; (b) OS survival curve of the two groups of patients.

**Table 1:** Baseline data of two groups of patients.

Baseline characteristic	Observation group (*n* = 55)	Control group (*n* = 45)	*p* value
Age, years old	57.14 ± 9.69	58.29 ± 10.39	0.635^a^
BMI (kg/m^2^)	22.06 ± 3.68	22.86 ± 3.08	0.526^a^
CEA (ng/mL)	6.13 (31.67)	4.36 (38.85)	0.320
Distance from the anus (mm)	46.69 ± 21.99	47.56 ± 21.04	0.927^a^
Diameter of tumor (mm)	51.20 ± 20.05	55.56 ± 19.62	0.295^a^
Gender			
Male	35	25	0.421^b^
Female	20	20	
Clinical T staging			
T2	11	7	0.843
T3	34	29	
T4	10	9	
Clinical N staging			
N0	9	9	0.348
N1	23	23	
N2	13	13	
Lateral pelvic lymph node metastasis			
Metastasis	14	18	0.136^b^
Nonmetastasis	41	27	

^a^Independent samples *t*-test. ^b^Fisher exact test. Double-tailed *p* values were used for all tests.

**Table 2:** Comparison of short-term efficacy of LARC patients receiving NAC with or without bevacizumab.

Preoperative baseline characteristics of TME	Observation group (*n* = 55)	Control group (*n* = 45)	*p* value
ypT staging			
T0	10	5	0.014
T1	9	7	
T2	20	6	
T3	16	25	
T4	0	2	
Total T downstaging	46	27	0.813^b^
ypN staging			
N0	46	33	0.080
N1	8	6	
N2	1	6	
Total N downstaging	42	30	0.813^b^

^b^Fisher exact test. Double-tailed *p* values were used for all tests.

**Table 3:** Perioperative complications of TME in the two groups.

Group	Anastomotic fistula	Early postoperative intestinal obstruction	Wound infection dehiscence	Urinary retention	Anastomotic bleeding	Total incidence
Control group (*n* = 45)	6	4	8	3	3	24
Observation group (*n* = 55)	2	1	3	2	2	10
*p* value	0.135^b^	0.171^b^	0.061^b^	0.655^b^	0.655^b^	<0.001^b^

**Table 4:** Adverse reactions of the two groups of patients during chemotherapy.

Group	Bone marrow suppression	Gastrointestinal reaction	Neurotoxicity	Leukopenia	Impaired liver and kidney function
Control group (*n* = 45)	16	26	13	22	14
Observation group (*n* = 55)	12	24	8	15	12
*p* value	0.179^b^	0.228^b^	0.090^b^	0.037^b^	0.361^b^

^b^Fisher exact test. Double-tailed *p* values were used for all tests.

## Data Availability

The data and materials in the current study are available from the corresponding author on reasonable request.
